This article has been retracted.

# Human Interferon Inducible Transmembrane Protein 3 (IFITM3) Inhibits Influenza Virus A Replication and Inflammation by Interacting with ABHD16A

**DOI:** 10.1155/2021/6652147

**Published:** 2021-03-03

**Authors:** Liang Chen, Limei Zhu, Jun Chen

**Affiliations:** ^1^Department of Infectious Diseases, Beijing Jishuitan Hospital, Beijing, China; ^2^Department of Chronic and Infectious Diseases Control, Jiangsu Provincial Center for Disease Control and Prevention, Nanjing, China; ^3^Department of Pathology, Nanjing Drum Tower Hospital, Nanjing, China

## Abstract

Studies have shown that human interferon inducible transmembrane protein (hIFITMs) family proteins have broad-spectrum antiviral capabilities. Preliminary studies in our laboratory have tentatively proved that hIFITMs have the effect of inhibiting influenza viruses. In order to further study its mechanism and role in the occurrence and development of influenza A, relevant studies have been carried out. Fluorescence quantitative polymerase chain reaction (PCR) detection technology was used to observe the effect of hIFITM3 on the replication of influenza A virus (IVA) and the interaction with hABHD16A. In HEK293 cells, overexpression of hIFITM3 protein significantly inhibited the replication of IVA at 24 h, 48 h, and 72 h; yeast two-hybrid experiment proved that hIFITM3 interacts with hABHD16A; laser confocal microscopy observations showed that hIFITM3 and hABHD16A colocalized in the cell membrane area; the expression level of inflammation-related factors in cells overexpressing hIFITM3 or hABHD16A was detected by fluorescence quantitative PCR, and the results showed that the mRNA levels of interleukin- (IL-) 1*β*, IL-6, IL-10, tumor necrosis factor- (TNF-) *α*, and cyclooxygenase 2 (COX2) were significantly increased. But when hIFITM3/hABHD16A was coexpressed, the mRNA expression levels of these cytokines were significantly reduced except COX2. When influenza virus infected cells coexpressing hIFITM3/hABHD16A, the expression level of inflammatory factors decreased compared with the control group, indicating that hIFITM3 can play an important role in regulating inflammation balance. This study confirmed that hIFITM3 has an effect of inhibiting IVA replication. Furthermore, it was found that hIFITM3 interacts with hABHD16A, following which it can better inhibit the replication of influenza virus and the inflammatory response caused by the disease process.

## 1. Introduction

Influenza virus is a representative strain of the Orthomyxoviridae family and includes human influenza virus and animal influenza virus (such as swine influenza virus, equine influenza virus, and avian influenza virus) [1]. There are four types of influenza viruses identified, namely, A, B, C, and D. Since the antigenicity of influenza A virus is extremely prone to mutation, it causes a high fatality rate in affected populations, is associated with rapid spread, and has been responsible for pandemics on multiple occasions; as such, it poses a serious challenge to medical communities as well as society as a whole. Due to the lack of drugs that are effective in treating such infectious diseases, outcomes and prognosis depend to a large extent on the elimination of pathogens by the body's own immune system [2].

Interferon-induced transmembrane proteins (IFITMs) are a class of host restriction factors that have been discovered in recent years. They can inhibit the proliferation of enveloped and nonenveloped viruses and are associated with a particular constitutive expression in a variety of cells [3]. It has been confirmed that IFITM3 can resist the infection of various viruses, including West Nile virus, influenza virus, and dengue fever. IFITM3 achieves an antiviral infection effect in a variety of ways [4, 5]. Studies on posttranscriptional modifications of IFITM3 have shown that IFITM3 can be modified by ubiquitination and palmitoylation, and these modifications regulate the cellular localization of IFITM3 and its antiviral function in different ways. Although research on the antiviral mechanism of IFITM3 has targeted the virus entry process, the specific mechanism is not yet clear.

Our preliminary research showed that overexpression of hlFITM3 significantly affected the replication of influenza virus. The purpose of this study was to further examine the anti-influenza virus effect of hlFITM3, its antiviral mechanism, and to inhibit the occurrence of inflammation during the replication of influenza virus with hlFITM3. A preliminary exploration of the mechanism was also conducted. The study of the hlFITM3 interacting protein and the regulation of this interaction in the inflammatory response caused by influenza virus infection can improve our understanding of the antiviral mechanism of IFITMs and provide a theoretical basis for the prevention and control of influenza.

## 2. Materials and Methods

### 2.1. Cell Culture

HEK293 cells were purchased from Shanghai Cell Bank, Chinese Academy of Sciences. All cells were grown in Dulbecco's modified Eagle's medium (DMEM) (Abcam, USA) with 10% fetal bovine serum and 1% antibiotics (penicillin and streptomycin). The cell culture was carried out in humidified air at 37°C containing 5% CO_2_. All cultures used standardized cell culture.

### 2.2. Construction of hlFITM3 Eukaryotic Expression Vector

After the total RNA of the cell was extracted, the first strand of cDNA was synthesized. The primers of the hABHD16A and hIFITM3 genes connected to the pEGFP-N1 vector and pCDNA3.1 vector are shown in Table 1.

Subsequently, the target gene was amplified, recovered, digested, ligated, and prepared for transformation to DH5a competent cells, and the recombinant plasmids were verified.

### 2.3. Plasmid Transfection

On the day before transfection, 2 × 10^5^ HEK293 cells were inoculated in a 6-well plate, with 2 mL of complete medium (without double antibodies) per well, and placed in a cell incubator, so that the cell density before transfection was about 60.70%. 4 *μ*g DNA and 8 *μ*L POLO deliverer 3000 were diluted in 50 *μ*L DMEM medium per well, mixed, and placed at room temperature for 5 min. The diluted solution of POLO deliverer 3000 was added dropwise to the diluted DNA solution, mixed gently, and left to stand at room temperature for 15 min. The above mixture was added dropwise to the cells in the 6-well plate and shaken gently. The transfected cells were cultured at 37°C and 5% CO_2_ for 48-72 h, and the medium was changed 12 h after transfection. 48 h after the completion of transfection, an inverted green fluorescence microscope was used to observe the expression of green fusion protein.

### 2.4. Viral Infection

On the day before transfection, 6 × 10^4^ cells were plated in a 24-well plate, and the positive plasmid carrying the target fragment was transfected into the cells. After 24 h of transfection, the complete medium was removed, 1x PBS was added, and the cell surface was washed 3 times. IVA diluent was added at 1 MOI (multiplicity of infection) and adsorbed in a 37°C and 5% CO_2_ incubator for 2 h. During this period, the samples were gently shaken every 30 min. After adsorption, the virus solution was removed, and 0.5 mL of DMEM complete medium containing 10% fetal bovine serum (FBS) was added to each 24-well plate and cultured at 37°C and 5% CO_2_. The culture supernatants were taken 24 h, 48 h, and 72 h after infection, and viral RNA was extracted according to the following viral RNA extraction (Takara Corporation, Japan) method.

### 2.5. Reverse Transcription-PCR (RT-PCR)

A PrimeScript miRNA RT kit (Takara Corporation, Japan) was used to reversely transcribe RNA into cDNA. RT-PCR was performed with a SYBR Green RT-PCR Kit (1 : 200, Takara Corporation, Japan). GADPH served as an internal control for RNA detection.

### 2.6. Western Blot

Proteins were extracted from cells using RIPA lysis buffer (Beyotime Biotechnology, China) containing protease inhibitors. A BCA protein detection kit was used for protein quantification. Protein separation was performed using 10% sodium dodecyl sulfate-polyacrylamide gel electrophoresis (SDS-PAGE). Then, the protein was transferred to a polyvinylidene fluoride (PVDF) membrane. The membrane was sealed with 5% skim milk. The membrane was subsequently incubated with the primary antibody (1 : 200) and then with the secondary antibody (1 : 2000). The antibodies used in this study were acquired from ABCAM, USA, and were subsequently tested to obtain images.

### 2.7. Statistical Processing

Statistical analysis was conducted using SPSS19.0 statistical software. Measurement data with a normal distribution and uniform variance were expressed as the mean ± standard deviation, and the univariate analysis of variance or repeated measurement was used to compare multiple groups of means, and the LSD *t*-test was used for further pairwise comparison. *P* < 0.05 was considered statistically significant.

## 3. Results

### 3.1. Construction of hlFITM3 Eukaryotic Expression Vector

Through gene cloning and vector construction, the results were verified by PCR and sequencing, and two types of eukaryotic fusion expression vectors pcDNA3.1-HA-hlFITM3 and pEGFP-N1-hlFITM3 were successfully constructed (Figures 1(a) and 1(b)).

The PCR results showed (Figure 1(c)) that the vectors used to knock out the hlFITM3 gene were constructed successfully: pHMG-hRNA-hhRNAlFITM3.

### 3.2. Overexpression of hlFITMs Has an Inhibitory Effect on Influenza Virus Replication

After transfecting HEK293 cells with pEGFP-N1-hlFITM3 and pcDNA3.1-HA-hlFITM3 for 24 h, they were infected with influenza virus at 1 MOI, and the culture supernatant was taken at different time points after infection. Fluorescence quantitative PCR was used to detect the virus copy number. The results showed that hIFITM3 had obvious anti-influenza virus effects. Virus amplification was significantly reduced at 24 h and 48 h after infection, when compared with controls. The difference became even more pronounced at 72 h (Figure 1(d)).

The constructed knockout plasmid was transfected into HEK293 cells, and a virus infection experiment was carried out. The results of fluorescence quantitative measurement showed that the pHMG-hRNA-hhRNAIFITM3 knockout plasmid was transfected, and the influenza virus infected the hlFITMl3 knockout cells. In contrast, the viral copy number was significantly increased (Figure 1(e)).

### 3.3. Subcellular Localization of hlFITM3 and hABHD16A

In the yeast transformation of hIFITM3 and hABHD16A, colonies grown on the SD-Leu-Trp solid medium lack leucine (Leu) and tryptophan (Trp), but in the lack of leucine (Leu), colonies were grown on pGBKT7-hIFITM3/pGADT7-hABHD16A on SD-Leu-Trp-His solid medium containing tryptophan (Trp) and histidine (His). It shows that hIFITM3 and hABHD16A can interact (Figure 2(a)).

The successfully constructed fusion fluorescent expression vector was transfected into HEK293 cells, and the pEGFP-N1/pdhRed-monomer-N1 empty vector was transfected as a control group. Hoechest33342 nuclear staining was performed and observed with a laser confocal microscope. The results showed that hlFITM3 and hABHDl6A were aggregated and localized in the cell membrane structure, respectively. The superimposed pictures show that hlFITM3 and hABHDl6A were colocated in the cell membrane structure (Figure 2(b)). After the plasmid was cotransfected for 24 h, the plasmid-transfected cells were infected with 1 MOI influenza virus, and culturing was continued for 48 h. They were subsequently stained by Hoechest33342 and observed by laser confocal microscopy. The results showed that after influenza virus infection, there was a clear change in the location of hlFITM3 and hABHDl6A as compared to before infection, and the colocalized area tended to move towards the cell's nuclear area.

### 3.4. hABHDl6A Has an Inhibitory Effect on IVA

The positive clones were verified by bacterial solution PCR, and the results showed that the pHMG-hRNA-hhRNAABHD16A was successfully constructed (Figure 3(a)). When hABHD16A was knocked out of HEK293 cells, the copy number of IVA increased significantly compared with the control, and the difference observed was significant. This result indicates that hABHD16A has an inhibitory effect on influenza A virus (Figure 3(b)). Once again, in HEK293 cells with an overexpression of hABHDl6A protein, there was no significant difference with the control group after 24 hours of infection with the virus. hABHDl6A affects IVA replication at 48 h after infection, which can also inhibit the replication of IVA virus at 72 h after infection (Figure 3(c)).

In HEK293 cells, when there was overexpression of hlFITM3 or hABHD16A alone compared to normal expressing cells, the results showed that hlFlTM3 significantly inhibited IVA replication at 24 h, 48 h, and 72 h after infection. When hABHD16A was overexpressed, it also significantly inhibited influenza virus replication at 24 h, 48 h, and 72 h after infection. After cotransformation of pcDNA3.1(+)-HA-hlFITM3/pcDNA3.1(+)-HA-hABHDl6A, the amount of virus that was detected at the three time points of infection showed that the inhibitory effect on coexpression of the two proteins against influenza virus was significantly stronger than when they were expressed alone. These findings show that hlFITM3 and hABHDl6A can synergistically inhibit the replication of influenza A virus (Figure 3(d)).

### 3.5. The Inhibition of IVA Replication by hlFITM3 Is Closely Related to the S-Palmitoylation of hABHDl6A

To determine whether the anti-influenza virus effect of hlFITM3 is related to its palmitoylation, PCR point mutation technology was used to amplify the palmitoylation site mutation (Figure 4(a)) and construct the mutant vector pcDNA3.1(+)-HA-hlFITM3-C50A-C5IA-C84A and pcDNA3.1(+)-HA-hlFITM3-C84A eukaryotic expression vector. M-hlFITM3, hlFITM3\hABHDl6A overexpressing hlFITM3, hABHDl6A, and C50A-C51A-C84A site mutations were infected with influenza A virus, and the culture supernatant was taken after 24 h, and the viral copy number was detected by RT-PCR. Compared with the transfection control group, after transfection of hlFITM3 and hABHDl6A and cotransfection of hlFITM3/hABHDl6A, the replication of influenza virus was significantly inhibited. In the cells transfected with mutant M-hlFITM3, the virus copy number was significantly higher than that in the wild transfected hlFITM3 group, and in cotransfected mutant M-hlFITM3\hABHDl6A, the virus copy number was higher than that of cotransfected hlFITM3/hABHDl6A. These results indicate that the antiviral effect of hIFITM3 depends on its palmitoylation site, and the function of this site is related to the hABHD16A interaction (Figure 4(b)).

### 3.6. Cotransfection of hlFITM3 and hABHDl6A Can Reduce the Expression of Inflammatory Factors Caused by IVA

Relative to uninfected cells, in flu virus-infected HEK293 cells, the hlFITM3 gene was significantly increased, and hABHDl6A gene expression was significantly reduced (Figures 5(a) and 5(b)).

When IL-6, TNF-*α*, IL-1*β*, and IL-10 were transfected with hlFITM3 and hABHDl6A, respectively, their expressions increased significantly, while with cotransfection, they decreased significantly, indicating that the interaction of hlFITM3 and hABHDl6A can reduce the expression of inflammatory factors. In the virus-infected group, the expression levels of IL6, TNF-*α*, IL-1*β*, and IL-10 were increased compared with the empty vector control, but the coexpression of hlFITM3 and hABHDl6A decreased IL-6, TNF-*α*, IL-1*β*, and IL-10 expression (Figures 5(d)–5(g)). In HEK293 cells, compared with control cells transfected with empty vectors, the expression level of the monocyte chemoattractant protein-1 (MCP-1) gene was significantly reduced in single transfection and cotransfection; in the infected virus group, the expression level of MCP-1 gene was lower (Figure 5(c)). The expression level of the COX2 gene was significantly increased when transfected with hlFITM3 and hABHDl6A as well as when cotransfected, respectively, while infection with influenza virus could reduce the expression level of COX2 (Figure 5(h)).

## 4. Discussion

This study confirmed that hIFITM3 has an effect of inhibiting IVA replication. Furthermore, it was found that hIFITM3 interacts with hABHD16A, following which it can better inhibit the replication of IVA and the inflammatory response caused by the disease process. The above results provide a possible explanation for the mechanism by which hIFITM3 inhibits the replication of IVA and offers theoretical support for clinically improving interferon to treat influenza infection.

Interferon-induced transmembrane proteins (IFITMs) are small transmembrane proteins induced by interferons (interferon, IFNs) [6]. Type I and type II interferons can induce the expression of human IFITM1, IFITM2, and IFITM3. As a specific viral restriction molecule, the virus is prevented from passing through the lipid bilayer of the cell and entering the cytoplasm. Human IFITM1, IFITM2, and IFITM3 are widely expressed in various tissues, and studies have found that IFITM3 is expressed in the upper respiratory tract and lung pleural cells. Interferon-induced transmembrane protein IFITM3 has a strong inhibitory effect on the replication of various viruses [7, 8]. IFITM3 is expressed on the cell membrane and exists on the cytoplasm as particles. IFITM3 plays a role in different cellular processes, including immune cell regulation, germ cell maturation, cell proliferation, and heart development [9, 10]. Influenza A virus is an RNA virus that is prone to mutation in the genome. The mutated virus exhibits increased infectivity, cross-species transmission and other phenomena, and even zoonotic conditions that threaten human health. Brass and Shapira and others first proposed IFITM3 as a potential limiting factor for IAV in 2009. Bailey et al. demonstrated that IFITM3-deficient mice not only failed to clear IAV but also found that there was an increase in the mortality rate after virus infection, as well as the risk of other diseases [11]. In terms of the mechanism of action, in their research, Huang et al. found that IFITM3 inhibits IAV infection by preventing the release of the riboprotein complexes about the cytoplasm, rather than through the inhibition of viral binding and entry into cells. Everitt et al. found that the single nucleotide polymorphism in the IFITM3 allele is related to the susceptibility to IAV [12, 13]. In addition, Gerlach et al. reported that the toxicity and spread of IAV are also related to the pH of the cell membrane and that the stable expression of IFITM2 and IFITM3 proteins can effectively reduce virus replication [14, 15]. In this study, influenza virus replication was inhibited from HEK293 cells overexpressing hlFITM3 protein. The virus was further suppressed via interaction with the protein hABHDl6A.

The ABHD protein family has now been predicted to contain at least 19 proteins [16]. This family of proteins has a typical domain of the *α*/*β*-hydrolase superfamily. The family contains proteases, lipases, esterases, dehalogenases, and peroxidases and oxide hydrolysis enzymes, etc. [17–19]. In the ABHD family, several members of the substrate have been identified as having the ability to regulate glycerophospholipid metabolism, and they may also play a role in lipid and energy metabolism [11, 20]. Therefore, this family of proteins has been described as potential regulators for lipid metabolism and signal transduction. The conserved structural motifs shared by these proteins suggest a synergistic role in lipid synthesis and degradation. The functional activity identification of the ABHD family has been reported, with the delineation of substrates and their connection to diseases that alter lipid metabolism in humans [21]. Existing predictions indicated that ABHD protein involves both hydrolase and acyl transferase activities. ABHD family proteins play an important role in physiological regulation, drug target screening, tumorigenesis, etc. Existing studies had indicated that ABHD is expected to become a new drug target. Among them, ABHD2 is predicted to have hydrolytic enzyme catalytic activity. Compared with wild-type mice, ABHD2 has been shown to be involved in smooth muscle cell migration and intimal thickening of vascular smooth muscle cells in homozygous mice [22]. Antisense oligonucleotides can be used to downregulate ABHD2 without affecting host cell physiology, blocking hepatitis B virus replication and expression. Indeed, the data indicate that this gene can be used as a new target for anti-HBV drug development. ABHD7 is predicted to negatively regulate the activity of epoxide lipids. Epoxy hydrolase 3 (EH3), or ABHD9, is associated with high expression levels in the skin and upper digestive tracts of mice. It is speculated that sEH inhibitors may be of value in the treatment of hypertension and type 2 diabetes. ABHD16A is a member of the *α*/*β*-hydrolase domain-containing (ABHD) family of metabolic serine hydrolases, also known as leukocyte antigen-B- (HLA-B-) related transcript 5 (HLA-B-associated transcript 5, BAT5) [23]. It has been reported that human ABHD16A is located on human chromosome 6 and has 21 exons and four transcripts. Existing studies had shown that the four transcripts contain two noncoding long-chain RNAs.

Protein palmitoylation is an important lipidation modification, which plays an important role in the transport of proteins, the location and function of organelles, cell signaling, metabolism, and the occurrence of apoptotic diseases and cancelation. Studies have shown that the S-palmitoylation site in the amino acid sequence of IFITM3 is essential for its function [24]. The results of this study on the anti-influenza virus effect of the mutants showed that after the corresponding mutation of the cysteine site, the effect of the virus was significantly weakened, similar to other reports related to IFITM3. Based on the results of subcellular localization, it has been speculated that this posttranslational S-palmitoylation modification may affect the binding of influenza virus to the membrane, as well as the separation, transport, and stability of membrane domains. This study also proved that hABHDl6A can effectively inhibit influenza virus and initially showed that it may interact with hlFITM3 to resist the possible mechanism of influenza virus replication.

This study also found that the expressions of hlFITM3 and hABHDl6A were significantly downregulated after the cells were infected with influenza virus, indicating that at the detected time point, the virus invasion led to changes in the expression of hlFITM3 and hABHDl6A, which suggests that these two genes may be involved in the regulation of virus invasion. However, whether downregulation of expression is due to immune escape of the virus needs further study. And at different time points of influenza virus invasion, the hABHDl6A gene was significantly reduced. After 48 hours of infection with influenza virus, it was found that hlFITM3 returned to a level close to that of the control group, which may indicate that the gene functions as the early stage of influenza virus invasion. In the early stage of influenza virus invasion (12 h), the expression levels of hlFITM3 and hABHDl6A genes were significantly increased, indicating an important suppression role in the process of influenza virus invasion. In this study, it was found that hlFITM3, as the main antiviral protein, was associated with significant biological activity in the process of virus invasion, which is consistent with previous research findings related to the antiviral effects of human IFITMs.

TNF-*α* is an important inflammation-related factor, which plays a key role in inflammation, autoimmunity, malignant tumor development, and apoptosis [25]. Existing research results indicate that influenza can cause elevated blood TNF-*α*, which has a discernible inhibitory effect on virus replication and, at the same time, recognizes the signals of the upstream cytokines IL-1 and IL-6, thus facilitating a response to sepsis caused by severe influenza [26, 27]. This study found that overexpression of hlFITM3 and hABHDl6A can promote significant expression of this cytokine. After overexpression of hlFITM3 and hABHDl6A in cells infected with influenza virus, it was found that the expression level of the factor was significantly reduced, further indicating that TNF-*α* is affected by influenza virus, and coexpression of both proteins led to a reduction in the level of TNF-*α*. IL-1*β* is a proinflammatory cytokine that can be expressed by many cell types and can be endogenous and competitive with IL-1 receptor antagonists (IL-IRA). Anti-inflammatory cytokines produced by tissues are suppressed.

IL-1*β* is an important proinflammatory cytokine of the innate immune response. After overexpression of hlFITM3, compared with the overexpression of influenza virus infection, IL-1*β* expression is significantly reduced. This is consistent with the results that IL-1*β* plays a key role in the inflammatory response by activating immune cells and inducing many secondary proinflammatory cytokines [28, 29]. The experimental results of this study indicate that overexpression of hlFITM3 and hABHDl6A can promote the expression of this cytokine, and the expression of this factor was not detected after cotransfection. Repeated experiments failed to detect presumed coexpression on multiple occasions. Later, mRNA levels were too low to be detected. Infected with influenza virus after coexpression, this factor was found to be upregulated. The results related to the effects of hlFITM3 and hABHDl6A on the expression of inflammatory factors suggest that the interaction of the two may play an important role in effectively balancing inflammation.

In conclusion, the research results obtained in this research broadened the antiviral spectrum of IFITM3, and the identification and function as its interacting proteins are expected to expand the direction of future research, to further explain the antiviral mechanism of IFITM3, with an analysis of the host cell in the defense against pathogenic microorganisms. The mechanism provides a strong theoretical research foundation. IFITM3 and ABHD16A may be used as new targets and potential antiviral factors in the future for the prevention and control of infectious diseases. Furthermore, future research on the anti-influenza mechanism of hlFITM3 and hABHDl6A will not only help to improve our understanding of innate immunity in the process of resisting the virus but also provide research ideas for the study about the resistance of other viruses.

## Figures and Tables

**Figure 1:** Construction of pEGFP-N1-hlFITM3 and pcDNA3.1-HA-hIFITM3 recombinant plasmids and anti-IAV detection of hIFITM3 in HEK293 cells. (a) Amplification of the target fragment of hIFITM3 (M: DM2000 DNA marker; hIFITM3: hIFITM3 PCR amplified fragment); (b) pEGFP-N1-hlFITM3 and pcDNA3.1-HA-hIFITM3 bacterial cell PCR (M: DM2000 DNA marker; pEGFP-N1-hlFITM3 and pcDNA3.1-HA-hIFITM3 PCR validation); (c) pHMG-hRNA-hhRNAIFITM3 (M: DM2000 DNA marker; pHMG-hRNA-hhRNAIFITM3: hhRNAIFITM3 knockout recombinant plasmids); (d) RT-PCR detection of IFITM3 (vs. control: ^∗^*P* < 0.05; ^∗∗^*P* < 0.01); (e) the effects on IAV replication of hIFITM3 knockout in HEK293 cells (vs. control: ^∗∗∗^*P* < 0.001).

**Figure 2:** Subcellular localization of hlFITM3 and hABHD16A. (a) Cotransfection of yeast two-hybrid screening. (b) Subcellular localization of hIFITM3 and hABHD16A in HEK293 cell (×400).

**Figure 3:** hABHDl6A has an inhibitory effect on influenza virus. (a) PCR validation of recombinant plasmid pHMG-hRNA-hhRNAABHD16A (M: DM2000 DNA marker; 1: pHMG-hRNA-hhRNAABHD16A); (b) the inhibition of IAV in HEK293 cells hABHD16A knockout (vs. control: ^∗^*P* < 0.05). (c) IAV copy number in hABHDl6A-overexpressing HEK293, at 24 h, 48 h, and 72 h (vs. control: ^∗^*P* < 0.05; ^∗∗^*P* < 0.01). (d) Effects of coexpression of hIFITM3 and hABHD16A on IAV replication (vs. pcDNA3.1 (+)-HA-hIFITM3: ^∗^*P* < 0.05; ^∗∗^*P* < 0.01; vs. pcDNA3.1 (+)-HA-hABHD16A: ^#^*P* < 0.05; ^##^*P* < 0.01).

**Figure 4:** (a) hIFITM3 mutant fragment PCR amplification (M: DM2000 DNA marker; l-4: hIFITM3-F, hIFITM3-R PCR amplification of the target fragment); (b) effects of coexpression of hIFITM3 and hABHDl6A on IAV replication (vs. 2: ^∗∗∗^*P* < 0.001; vs. 5: ^##^*P* < 0.01). 1: vector; 2: overexpression hIFITM3; 3: overexpression hABHDl6A; 4: overexpression of hIFITM3 with mutations at 50A-C51A-C84A; 5: overexpression hIFITM3/hABHD16A; 6: overexpression of hIFITM3/hABHDl6A with mutations at 50A-C51A-C84A.

**Figure 5:** Effect of hIFITM3 and hABHDl6A on the expression of inflammatory factors. (a) hIFITM3 expression levels after IAV infection (vs. mock: ^∗^*P* < 0.05, ^∗∗^*P* < 0.01, and ^∗∗∗^*P* < 0.001). (b) hABHD16A expression after IAV infection (vs. mock: ^∗^*P* < 0.05, ^∗∗^*P* < 0.01, and ^∗∗∗^*P* < 0.001). (c–h) Effects on the expression of inflammatory factors (MCP-1, IL-6, TNF-*α*, IL-1*β*, IL-10, and COX2) after overexpression of hIFITM3 and/or hABHDl6A in HEK293 cells (vs. vector: ^∗^*P* < 0.05, ^∗∗^*P* < 0.01, and ^∗∗∗^*P* < 0.001). 1: hIFITM3; 2: hABHDl6A; 3: hIFITM3/hABHDl6A; 4: hIFITM3 (IAV); 5: hABHDl6A (IAV); 6: hIFITM3/hABHDl6A (IAV).

**Table 1:** The sequence of the primers.

	Gene	The sequence of the primers
pEGFP-N1:ABHDl6A	F	5′-primer CGGAATTCATGGCGAAGCTGCTG
	R	3′-primer CGGGATCCAGGTGCCAGGGCAT
pEGFP-N1:IFITM3	F	5′-primer ACGGAATTCATGAATCACACTGTCCAA
	R	3′-primer CGGGATCCCTTCCATAGGCCTGGAAGA
pCDNA3.1:ABHDl6A	F	5′-primer CGGAATTCATGGCGAAGCTGCTG
	R	3′-primer CGGGATCCAGGTGCCAGGGCAT
pEGFP-N1:IFITM3	F	5′-primer CGGAATTCATGAATCACACTGTCCAA
	R	3′-primer CGGGATCCCTTCCATAGGCCTGGAAGA

## Data Availability

The data used to support the findings of this study are available from the corresponding author upon request.
